# An Artificial Intelligence-Based Reactive Health Care System for Emotion Detections

**DOI:** 10.1155/2022/8787023

**Published:** 2022-05-18

**Authors:** Gouse Baig Mohammad, Sirisha Potluri, Ashwani Kumar, Ravi Kumar A, Dileep P, Rajesh Tiwari, Rajeev Shrivastava, Sheo Kumar, K. Srihari, Kenenisa Dekeba

**Affiliations:** ^1^Department of Computer Science and Engineering, Vardhaman College of Engineering, Hyderabad, India; ^2^Department of CSE, Faculty of Science and Technology-IcfaiTech, The ICFAI Foundation for Higher Education, Donthanapally, Shankarpalli Road, Hyderabad, Telangana 501203, India; ^3^Head Department of CSE (AIML) and Professor, Sreyas Institute of Engineering and Technology, Hyderabad, India; ^4^Department of Computer Science Engineering, Sridevi Women's Engineering College, Gandipet, India; ^5^Department of Computer Science and Engineering, Malla Reddy College of Engineering and Technology, Kompally, Hyderabad, India; ^6^CMR Engineering College, Hyderabad, India; ^7^Department of ECE, Princeton Institute of Engineering and Technology for Women, Hyderabad, India; ^8^CMR Engineering College, Hydrabad, India; ^9^Department of Computer Science and Engineering, SNS College of Technology, Coimbatore, India; ^10^Department of Food Process Engineering, College of Engineering and Technology, Wolkite University, Wolkite, Ethiopia

## Abstract

In the past few years, remote monitoring technologies have grown increasingly important in the delivery of healthcare. According to healthcare professionals, a variety of factors influence the public perception of connected healthcare systems in a variety of ways. First and foremost, wearable technology in healthcare must establish better bonds with the individuals who will be using them. The emotional reactions of patients to obtaining remote healthcare services may be of interest to healthcare practitioners if they are given the opportunity to investigate them. In this study, we develop an artificial intelligence-based classification system that aims to detect the emotions from the input data using metaheuristic feature selection and machine learning classification. The proposed model is made to undergo series of steps involving preprocessing, feature selection, and classification. The simulation is conducted to test the efficacy of the model on various features present in a dataset. The results of simulation show that the proposed model is effective enough to classify the emotions from the input dataset than other existing methods.

## 1. Introduction

Affective communication is essential in many fields, including public health, crisis response, and feedback analysis, to name just a few [1]. Emotions in humans can be expressed vocally, through text or through physical sensations. Humans are capable of recognising a wide range of emotions and thoughts, but computers are unable to distinguish between the intensity and emotion. In the field of research, emotion analysis is a prominent topic since it provides a means of communicating with machines [2].

Despite the fact that researchers have put a lot of effort into text-based emotion recognition, the applications are diverse. In accordance with the literature, textual data, which include social media content and discussion communities, are the primary source of emotion detection [3]. Based on health data, it is also beneficial to distinguish between positive and negative emotions based on health data because unpleasant emotions can be harmful and can result in risky mental or physical states of mind. People emotional well-being is modified when they suffer from depression, anxiety, loneliness, and other mental health problems. As a result of this development, the area of psychology is in desperate need of research into the identification and mapping of emotions in text [4].

Because emotions and feelings are not described in the literature, there is no general agreement. What we call feelings are sometimes underappreciated in and of themselves, since they are frequently characterised in terms such as outrage and nausea [5]. It is possible to experience rapid and frequent changes in mood while unwell. We can observe or communicate our interior states through many means, but this depiction is devoid of intellect and meaning. A behaviour that involves extremely complex components, data from a diverse variety of sources, and evidence gathered over a longer period of time, on the contrary, is in opposition to this [6].

As an example, happy or joy is one of the enthusiastic states that can be attained by experiencing typically positive feelings. When a guy is in excellent health, his emotions tend to be more optimistic, and when in poor health, his emotions tend to be more depressed [7]. When people are sick, they experience feelings of unpleasantness, grief, and disappointment, and these feelings can lead to suicidal ideation in the most extreme cases if the disease lasts for an extended period of time. As part of our research, we gathered information about patient emotions from a variety of disease-related news pieces that were posted on a variety of websites [8, 9].

The keyword-based strategy is the most widely used and straightforward method available. This technique searches for the emotive term in the sentence and then a matching pattern is applied in order to extract the keyword [10]. Natural language processing (NLP) techniques can be used to tokenize text, and the intensity of words can also be calculated using these techniques. On the contrary, the Lexicon method uses lexicons to determine the emotions present in a piece of textual material [11]. This approach determines if a keyword has a positive or negative meaning based on the probability of its occurrence. The main problem in this existing scenario is to gather information about patient emotions from a variety of disease-related news pieces that were posted on a variety of websites.

The main contribution in this study is mentioned below:

- An artificial intelligence-based classification that aims to classify the emotions from the input data using metaheuristic feature selection and machine learning classification.
- The proposed model is made to undergo series of steps involving preprocessing, feature selection, and classification.
- In the feature selection, the proposed Intelligent Water Drop algorithm is included in the proposed system as a classifier. With the help of an Intelligent Water Drop algorithm, selecting the greatest characteristics or qualities that are near to the best is straightforward.

## 2. Related Works

By the time, artificial intelligence (AI) became popular; machine learning had already provided some of the most innovative solutions to a wide range of issues, including breakthroughs in linguistics and NLP methodologies [12]. Emotions derived from sentences are classified using a number of algorithms in the field of computer science. Aside from that, researchers employed the lexicon-based approach to predict election results based on the categorization of emotions in Twitter data [13].

Emotional iconography, as well as the written word, is used by the authors in [14] to determine the feelings of their readers. They employ a range of methodologies in their work, including keyword analysis, as well as keyword negation analysis, as well as a collection of proverbs and emoticons. Their calculations show that their approach has a success rate of 87%, which is very high. Several studies in the literature have used NLP approaches to create handwritten dictionaries of common expressions [15].

Several studies on the subject of research have looked into the ways in which writing might convey feelings. Big data were used by the authors in both [16, 17], as well as in other publications. In a separate study [17], the potential of machine learning algorithms to effectively recognise emotions in Internet material was investigated. The results were promising.

In [18], a summary of the datasets and approaches available for emotion analysis is described in detail. According to their research, emotion-labeled datasets are hard to come by and are not available to the general public for use. Third-party APIs are used in many studies on the classification and detection of emotions in text, which is why they are so popular. Sentiment analysis is two of the most frequently encountered applications of the application programming interface (API). Other applications include the identification of malicious intent and the recognition of abusive text.

## 3. Proposed Method

The proposed model, which is shown in Figure 1, is made to undergo series of steps involving preprocessing, feature selection, and classification.

### 3.1. Preprocessing

We begin by purifying the data in order to achieve the best results. The use of simple preprocessing techniques such as lowercase conversion, punctuation removal, and stop word removal can help us improve the quality of our output. The steps for text cleaning are detailed in greater detail below.

#### 3.1.1. Lowercase Conversion

Lower case conversion is the first step in the preprocessing process. The text is changed to lower case in order to prevent duplicates from being created when the database is cleaned. In spite of the fact that the terms happy and happy are spelled differently, they are treated as separate words due to differences in case usage. We employ the lower case conversion approach in order to avoid confusion.

#### 3.1.2. Punctuation Removal

It is required to eliminate all punctuation from the text in order for the model to be trained more effectively. All punctuation occurrences should be removed from the text dataset in order to assist the model in acquiring functional attributes rather than nonfunctional properties.

#### 3.1.3. Removal of Stop Words

Stop words are prior training the machine learning model because they do not provide much context for the text data. Here, the nltk.corpus module in Python is useful because it contains stop words in the English language.

#### 3.1.4. Common Words' Removal

It is standard practise to exclude terms from a corpus if they are too similar to one another. Incorporating overlap in vocabulary into machine learning classifiers' evaluation scores has a negative impact on the results. Due to the fact that their inclusion will have no impact on our text classification, these terms have been omitted.

#### 3.1.5. Rare Words' Removal

In the same way that we deleted the most frequently recurring terms from the text, we also eliminated the terms that appeared just once or twice in the text. Despite the fact that they are extremely rare, noise tends to overshadow their significance.

#### 3.1.6. Resampling

Table 1 indicates unequivocally that the distribution of emotion classes is not uniformly distributed across the board. When dealing with uneven data, data resampling becomes important. When executing a resampling procedure on a dataset, it is possible to over- or under-sample the dataset. The data are resampled to ensure that both the majority and minority classes are taken into consideration.

After the data have been appropriately balanced, the analysis is carried out from two perspectives, namely, including and excluding the minority class, respectively.

### 3.2. Feature Selection Using Intelligent Water Drop Algorithm

It is possible to lower classification error rates while also achieving the best results by selecting the best features from a huge dataset.

Intelligent Water Drop algorithm is included in the proposed system as a classifier. With the help of an Intelligent Water Drop algorithm, selecting the greatest characteristics or qualities that are near to the best is straightforward. The work flow of Intelligent Water Drop is determined by the riverbed, the soil, and the drop velocity (features):

(1) $$\begin{array}{c} \text{velocity}\left(t+1\right)=\text{vel}\left(t\right)+\left(\frac{q}{b_{v}+c_{v}*{\text{soil}}^{2a}\left(I,j\right)}\right), \end{array}$$

where velocity (*t* + 1) = velocity of particles, *b*_*v*_ and *c*_*v*_ denote static, and *q* denote dynamic parameters.

When using this approach, the best feature is computed by taking into account both static and dynamic characteristics. The static parameters, in contrast to the dynamic parameters, remain constant during the entire procedure, whereas the dynamic parameters change. The Intelligent Water Drop feature selection process begins with the aid of a graph, and the features are dispersed throughout the search area to aid in the process. When the static parameter is determined, the dynamic parameters, velocity, and soil properties are calculated from it, and the values are updated accordingly.

There is a repeating procedure for all of the features, which aids in the identification of the overall solution. A consequence of this is that the abovementioned updating approach gives the attributes that are most relevant for the future categorization stage.

### 3.3. Classification Using BPNN

According to the researchers (Patterson, 1996), ANNs trained on data from real-world datasets have been successful at projecting the level of a specific event outcome. There have been numerous studies showing that artificial neural networks outperform more traditional statistical pattern detection techniques. For this purpose, it was decided to use a three-layer BPNN structure to estimate the features.

There was a significant amount of features present, which corresponded to the values that were entered. The root mean square error (RMSE) was employed for the purposes of training, validation, and testing. The RMSE was used to determine the ideal number of concealed nodes. The RMSE for the testing set will be calculated by selecting the best hidden nodes.

  Step 1: the outputs of the first phase (forward propagation) are calculated depending on the values of the inputs and the weights that are currently in effect. There are several factors that influence the net excitation of each hidden unit and output unit. These include: unit values from earlier layers that are associated with the unit at issue. This function determines the relative relevance of one unit of measurement in comparison to another.

Upon completion of the activation function, the calculated output value for that unit based on this net excitation is returned. It is necessary to have an activation function that is both continuous and differentiable. In BPNN, a number of activation functions can be used to achieve the desired result. The activation function sigmoid is one of the most commonly used.

  Step 2: it is possible to estimate the backward propagation of error by comparing the output of the target to the output of each output unit, which is then multiplied by the total number of output units. This mistake has been forwarded to the preceding layer, which is currently hidden. For each unit, the error in the hidden layer *N* is defined by a mathematical formula. *N*−1 is the previous hidden layer, and the errors are calculated in a similar manner at each node of *N*−1, the previous hidden layer. Correcting the weights based on the determined errors reduces the error at each output unit to the bare minimum. When errors are repeated in both the forward and backward directions, they are decreased to the desired level.

## 4. Results and Discussion

In this section, we discuss the text emotional dataset for detecting the emotional states in patients based on their textual interactions with the researchers. Currently, there is no comprehensive dataset for the automatic emotion recognition in patients via text, as far as we are aware. This work proposes EmoHD as a new standard for the automatic emotion recognition in text data. Using a dataset such as Fer2013, it is possible to detect or recognise facial expressions.

It is necessary, however, for the advancement of research in this sector that the ability to recognise emotions in patients relevant to diseases be mastered (Table 2). The study believes that the following four qualities should be included in every database of healthcare-related news. It is critical to have large samples in each class, as well as an appropriate value assigned to each emotion.

Figure 2 shows the results of accuracy on test dataset (20%) of the entire dataset and the results of simulation shows that the proposed method achieves higher rate of accuracy than BPNN, ANN, MLP, and RBF.

Figure 3 shows the results of specificity on test dataset (20%) of the entire dataset and the results of simulation shows that the proposed method achieves higher specificity than BPNN, ANN, MLP, and RBF.

Figure 4 shows the results of sensitivity on test dataset (20%) of the entire dataset and the results of simulation shows that the proposed method achieves higher sensitivity than BPNN, ANN, MLP and RBF.

Figure 5 shows the results of F-measure on test dataset (20%) of the entire dataset and the results of simulation shows that the proposed method achieves higher F-measure than BPNN, ANN, MLP, and RBF.

As a result of this technology, it becomes possible to recognise or identify the patient real-time mental state while he or she is receiving treatment. It is necessary to have an emotion-labeled dataset in order to detect emotion in text data from a patient who is suffering from a medical condition. A dataset that has been emotionally labeled and is scattered over a variety of diseases is therefore critically required in this context.

## 5. Conclusions

In this study, we develop an intelligent water drop-based artificial neural network classification system that aims to detect the emotions from the input data using metaheuristic feature selection and machine learning classification. The proposed model is made to undergo series of steps involving preprocessing, feature selection, and classification. The simulation is conducted to test the efficacy of the model on various features present in a dataset. The results of simulation show that the proposed model is effective enough to classify the emotions from the input dataset than other existing methods. From the results, it is seen that the proposed intelligent water drop-based artificial neural network classification attains a classification rate of 90% than the other existing methods. In future, the accuracy and classification rate can be improvised with some more deep learning algorithms.

## Figures and Tables

**Figure 1:** Proposed method.

**Figure 2:** Accuracy on test dataset.

**Figure 3:** Specificity on test dataset.

**Figure 4:** Sensitivity on test dataset.

**Figure 5:** F-measure on test dataset.

**Table 1:** Emotion class label.

Emotion class	Count
**Angry**	1343
**Sad**	358
**Fear**	742
**Excited**	1215
**Bored**	22
**Happy**	522

**Table 2:** Overall features on EmoHD dataset.

Features	Count
Number of words	1634319
Characters	12090922
Numerics	64543
Unique trigrams	1159467
Unique bigrams	827475
Unique unigrams	91988

## Data Availability

The datasets used and/or analyzed during the current study are available from the corresponding author uon reasonable request.
